The article "TFEB-NF-κB inflammatory signaling axis: a novel therapeutic pathway of Dihydrotanshinone I in doxorubicin-induced cardiotoxicity" was published in 2020. Journal: J Exp Clin Cancer Res.

# TFEB-NF-κB inflammatory signaling axis: a novel therapeutic pathway of Dihydrotanshinone I in doxorubicin-induced cardiotoxicity

**DOI:** 10.1186/s13046-020-01595-x

**Published:** 2020-05-24

**Authors:** Xiaoping Wang, Qiyan Wang, Weili Li, Qian Zhang, Yanyan Jiang, Dongqing Guo, Xiaoqian Sun, Wenji Lu, Chun Li, Yong Wang

**Affiliations:** 1 School of Life Science, Beijing University of Chinese Medicine, Beijing, 100029 China; 2 School of Traditional Chinese Medicine, Beijing University of Chinese Medicine, Beijing, 100029 China; 3 Modern Research Center for Traditional Chinese Medicine, Beijing University of Chinese Medicine, Beijing, 100029 China

**Keywords:** TFEB-NF-κB, Inflammation, Doxorubicin, Cardiotoxicity, Dihydrotanshinone I

## Abstract

**Background:**

Doxorubicin is effective in a variety of solid and hematological malignancies. Unfortunately, clinical application of doxorubicin is limited due to a cumulative dose-dependent cardiotoxicity. Dihydrotanshinone I (DHT) is a natural product from Salvia miltiorrhiza Bunge with multiple anti-tumor activity and anti-inflammation effects. However, its anti-doxorubicin-induced cardiotoxicity (DIC) effect, either in vivo or in vitro, has not been elucidated yet. This study aims to explore the anti-inflammation effects of DHT against DIC, and to elucidate the potential regulatory mechanism.

**Methods:**

Effects of DHT on DIC were assessed in zebrafish, C57BL/6 mice and H9C2 cardiomyocytes. Echocardiography, histological examination, flow cytometry, immunochemistry and immunofluorescence were utilized to evaluate cardio-protective effects and anti-inflammation effects. mTOR agonist and lentivirus vector carrying GFP-TFEB were applied to explore the regulatory signaling pathway.

**Results:**

DHT improved cardiac function via inhibiting the activation of M1 macrophages and the excessive release of pro-inflammatory cytokines both in vivo and in vitro. The activation and nuclear localization of NF-κB were suppressed by DHT, and the effect was abolished by mTOR agonist with concomitant reduced expression of nuclear TFEB. Furthermore, reduced expression of nuclear TFEB is accompanied by up-regulated phosphorylation of IKKα/β and NF-κB, while TFEB overexpression reversed these changes. Intriguingly, DHT could upregulate nuclear expression of TFEB and reduce expressions of p-IKKα/β and p-NF-κB.

**Conclusions:**

Our results demonstrated that DHT can be applied as a novel cardioprotective compound in the anti-inflammation management of DIC via mTOR-TFEB-NF-κB signaling pathway. The current study implicates TFEB-IKK-NF-κB signaling axis as a previously undescribed, druggable pathway for DIC.

## Background

Doxorubicin (DOX) is one of the most commonly used chemotherapeutic drugs for a wide range of cancers, such as leukemia, soft tissue sarcomas and breast cancer [1]. However, the rate of DOX-induced cardiotoxicity (DIC) is reported to be as high as 57%, and the mortality rate from these heart diseases is reported to be 8.2 times higher than that in healthy people [2]. Currently, dexrazoxane is the only FDA approved drug for the protection against cardiotoxicity. However, the Committee for Medicinal Products for Human Use (CHMP) in the UK has published the outcome of a referral that recommends several restrictions on dexrazoxane use in both children and adults with cancer. Therefore, there is an urgent need to identify the underlying mechanism of DIC and novel therapeutic agents that can prevent and/or reverse DOX-induced cardiovascular adverse effects. Recently, inflammation induced by doxorubicin has been identified as a high risk factor for developing heart failure and drugs with anti-inflammatory properties are attractive therapeutics for alleviating DIC [3, 4].

The article "TFEB-NF-κB inflammatory signaling axis: a novel therapeutic pathway of Dihydrotanshinone I in doxorubicin-induced cardiotoxicity" was published in 2020. Journal: J Exp Clin Cancer Res.

Nuclear factor-κB (NF-κB)-mediated inflammatory pathway is a classic signaling cascade that controls the expressions of pro-inflammatory genes in multiple types of cells. In the resting state, inactive NF-κB is sequestered in the cytoplasm by IκB (inhibitor of NF-κB). Under stimulation of pro-inflammatory signals, IKKs (IκB kinases) are activated which phosphorylates IκB on serine residues. Phosphorylated IκB will be degraded and active NF-κB dimers will be released and translocated into nucleus, inducing expressions of inflammatory cytokines, such as tumor necrosis factor-α (TNF-α) and interleukin 8 (IL-8). Several studies have confirmed that levels of inflammatory cytokines are increased in myocardial cells under doxorubicin-stimulated condition [5, 6]. Furthermore, hyper-activation of NF-κB is implicated in inflammatory responses in DIC [5, 7]. Nevertheless, the regulatory mechanisms of NF-κB transcriptional activity in DIC are still unclear.

The mammalian target of rapamycin (mTOR) is an atypical serine/threonine kinase, which regulates physiological homeostasis at the cellular and holistic level. Transcription factor EB (TFEB) plays a master role in governing basic cellular processes [8]. The mTOR-mediated phosphorylation negatively regulates TFEB nuclear translocation and activity [9]. It is of note that rapamycin analogues are therapeutically used as immuno-suppressants, and TFEB was also validated to have potential anti-inflammatory effect [10]. In this study, we further investigated whether mTOR-TFEB pathway plays a role in DIC-related inflammation. A profound understanding of this mechanism will provide a basis for discovery of novel targets as well as the therapeutic agents in alleviating DIC.

The article "TFEB-NF-κB inflammatory signaling axis: a novel therapeutic pathway of Dihydrotanshinone I in doxorubicin-induced cardiotoxicity" was published in 2020. Journal: J Exp Clin Cancer Res.

Salvia miltiorrhiza Bunge has been widely applied in traditional Chinese medicine (TCM) for a long history in the treatment of various inflammatory diseases [11]. As a dietary supplement, it is the first TCM to be documented in USP 37-NF32. Dihydrotanshinone I (DHT) is the one of major active diterpenes in the liposoluble extract [12]. Studies have shown that DHT possesses a variety of anti-tumor and anti-inflammatory properties [13–16]. However, whether DHT could alleviate DIC and whether the protective effect is medicated by the anti-inflammatory pathway remain elusive. In this study, we established an in vitro DOX-stimulated H9C2 model and an in vivo DIC mice model. The anti-inflammatory mechanism of DHT was investigated. This study will provide insight into the anti-inflammatory strategies and drug combination therapy in the management of DIC.

## Methods

### Reagents and chemicals

Saline was purchased from SiYao Co., Ltd. (Shijiazhuang, China). Doxorubicin was bought from ApexBio Technology LLC (Houston, TX, United States). DHT was purchased from Shanghai Shidande SDHTdard Technical Service Co., Ltd. (Shanghai, China). Rapamycin was purchased from Sangong Pharmaceutical Co., Ltd. (Shanghai, China). 4% paraformaldehyde was from Beijing Applygen Technology Inc. (Beijing, China). Dimethyl sulfoxide (DMSO) was purchased from Sigma-Aldrich LLC (Shanghai, China). PDTC was purchased from Abmole China Branch. MHY1485 was purchased from Selleck (Houston, TX, United States). Dulbecco’s Modification of Eagle’s Medium (DMEM), Fetal Bovine Serum (FBS), Penicillin, streptomycin, 0.1 mol/L sodium cacodylate buffer, sodium carboxymethylcellulose and DAPI were purchased from Beijing BioDee Biotechnology Co., Ltd. (Beijing, China). GFP-TFEB lentiviral vector were bought from Hanbio Technology Co., Ltd. (Shanghai, China). All other chemicals were purchased from commercial sources.

### Establishment of DIC model in Zebrafish, *in mice and pharmacological treatments*

The DIC model in zebrafish was established according to the methods described in a previous study [17]. Briefly, after the heart had formed and circulation had begun 1 day postfertilization (dpf), zebrafish were treated with 100 μM DOX or/and 10 nM DHT, and phenotypic changes, including fraction shortening (FS), the blood speed of the tail vein, heart rate and survival rate were respectively assessed at three dpf.

C57BL/6 male mice (18 g ± 2 g) were purchased from Beijing SPF Biotechnology Co., Ltd., China (Beijing, China). All mice were housed at temperature 22 ± 2 °C, with proper humidity, lighting (12 h light/12 h dark cycle), and free access to food and water. All mice were randomized into four groups as follows: 16 mice in the DOX group, DHT-treated group or positive drug (Rapamycin, Rapa)-treated group, respectively; 10 mice in Saline group. DIC model was induced via tail vein injection with DOX (5 mg·kg^− 1^) once weekly for 4 weeks and sham group was given with saline (0.9% NaCl) at the same time. This mice model has been described in previous study [18]. Besides, as the positive control drug, Rapamycin, an inhibitor of mTOR, was widely reported to be able to alleviate cardiac inflammation [19, 20]. Each drug was orally and daily administered for 4 weeks starting on 1 week after the last DOX injection. The doses of DHT (20 mg·kg^− 1^) and Rapamycin (2.81 mg·kg^− 1^) were determined based on previous studies [21, 22]. Given that DHT and Rapamycin are both poorly soluble in water, we applied 0.5% aqueous solution of a sodium carboxymethylcellulose (CMC) as the suitable vehicle as previous literature described. And the Saline group and the DOX group received the same volume of vehicle. All animal procedures were carried out in accordance with the Guide for the Care and Use of Laboratory Animals (NIH Publications No.85–23) and with Beijing University of Chinese Medicine Animal Care Committee (approve code BUCM-4-2,018,101,504-4068). After study, all mice were anaesthetized by isoflurane inhalation 2% and then euthanized by cervical dislocation.

The article "TFEB-NF-κB inflammatory signaling axis: a novel therapeutic pathway of Dihydrotanshinone I in doxorubicin-induced cardiotoxicity" was published in 2020. Journal: J Exp Clin Cancer Res.

### Echocardiographic assessment of cardiac functions

After 4 weeks’ administration, cardiac function was examined by Transthoracic echocardiography (Vevo TM 2100; Visual Sonics, Canada). Left ventricular end-diastolic volume (LVEDV), left ventricular end-systolic volume (LVESV), left ventricular end-diastolic dimension (LVEDD) and left ventricular end-systolic dimension (LVESD) were assessed for at least three uninterrupted cardiac cycles. Then mice were sacrificed, heart and blood were collected.

### Histological examination

For histological analysis, hearts were immersed in 4% paraformaldehyde for at least 24 h, then were embedded in paraffin and cut into 4 μm serial slices. Paraffin sections were stained with Hematoxylin-Eosin (HE) and were monitored under an optical microscope at 400 × magnification.

### Malondialdehyde (MDA) assay and superoxide dismutase (SOD) assay

MDA and SOD content commonly reflect the level of oxidative stress. Evidences showed that oxidative stress and inflammation are regarded as essential partners presenting simultaneously and interact with each other in diverse pathological conditions. MDA content and SOD activity in plasma were detected by following the instructions of commercially available kits (Jiancheng, Nanjing, China). MDA level was expressed as nmol/L in plasma. SOD activity was expressed as U/mL in plasma.

The article "TFEB-NF-κB inflammatory signaling axis: a novel therapeutic pathway of Dihydrotanshinone I in doxorubicin-induced cardiotoxicity" was published in 2020. Journal: J Exp Clin Cancer Res.

### Immunochemistry

The slices were dewaxed with xylene and gradient alcohol hydration, then were added with drops of 3% H_2_O_2_ for resting 15 min to block endogenous peroxidase. After washing with phosphate buffered saline (PBS) for three times, the cartilage slices were added with heated sodium citrate buffer for microwaving 6 min to antigen repair, which was repeated twice. After cooling and washing with PBS, the cartilage slices were treated with 5% goat serum for 10 min, to obstruct the binding of nonspecific antibody, then added with drops of the first antibodies of TNF-α. Later the slices were incubated at 37 °C for about 30 min and washed with PBS. After reacting with the second antibody, the slices were incubated at 37 °C for another 30 min and washed with PBS, later followed by staining for 10 min with diaminobenzidine (DAB), washing with running pure water, re-staining with hematoxylin and mounting with neutral balsam. Finally, we observed the images under a microscope and picture-taking.

### Flow cytometry

Flow cytometry was performed referring to literature concerned [23]. Hearts from mice (three mice per group) were minced into small pieces around 1 mm^3^ followed by digestion with 40% collagenase II (17101–015; Invitrogen, CA, United States) and 0.25% Trypsin (17104–019; Invitrogen, CA, United States) for 10 min. To disperse solid tissue into single cells, the enzymes (mainly collagenase and protease) were used to digest collagen fibers and elastic fibers, and to hydrolyze proteins and mucopolysaccharide substances that tight junction structure of tissue cells [24, 25]. Then cells were put into centrifuge at a force of 300 g for 5 min. After washing two times with PBS, cells were resuspended with 200 μL PBS, then stained with 0.75 μg anti-CD11b, 1 μg anti-F4/80, 1 μg anti-CD86 and 1 μg anti-CD206 antibodies. Followed by examining on a FACS Canto II flow cytometer (BD Biosciences). Data were analyzed by using the FlowJo software (FlowJo, LLC, Ashland, OR, USA). The antibodies were listed in Table 1.

**Table 1:** Antibodies used in Flow cytometry

Protein	Antibody
PE-Cy7 Rat Anti-CD 11b Clone M1/70	561,098; BD PMG, United States
F4/80 (BM8.1) Rat mAb (APC Conjugate)	86,007; Cell Signaling Technology, Germany
PE anti-mouse CD86	105,105; BioLegend, United States
FITC anti-mouse CD206 (MMR) Antibody	141,703; BioLegend, United States

### Establishment of LPS-induced RAW264.7 cell model and pharmacological treatments

RAW 264.7 macrophages in our study were obtained from China Infrastructure of Cell Line Resources. RAW 264.7 macrophages were cultured in DMEM supplemented with 10% FBS at 37 °C in a humidified atmosphere (5% CO_2_ and 9% O_2_). To evaluate the effects of DHT on LPS-induced RAW264.7, cells were stimulated with LPS (1 μ g/mL) for 24 h with or without DHT (added to media 2 h before treating with LPS). The concentrations of DHT in culture media in different cell groups were 10, 50 and 100 nM, respectively.

The article "TFEB-NF-κB inflammatory signaling axis: a novel therapeutic pathway of Dihydrotanshinone I in doxorubicin-induced cardiotoxicity" was published in 2020. Journal: J Exp Clin Cancer Res.

### Detection for TNF-α in the supernatant

Cell supernatants were collected from LPS-induced RAW 264.7 (with or without DHT pretreatment). The concentrations of TNF-α and IL-1β in the supernatants were determined by using ELISA kits bought from Boster Biological Technology co.ltd and the manufacturer’s instructions were followed. TNF-α and IL-1β levels were expressed as pg/mL.

### Establishment of DOX-stimulated H9C2 cell model and pharmacological treatments

H9C2 cells in our study were obtained from China Infrastructure of Cell Line Resources. The establishment of DOX-stimulated H9C2 cell model has been mentioned in our previous study [26]. For pharmacological treatments, we set up various groups: Control group, DOX group (with DOX 1 μM), DOX + DHT group (with DHT 10 nM), DOX + DHT + MHY1485 group (with DHT 10 nM and MHY1485 5 μM) and DOX + PDTC group (with PDTC 100 nM). For western blot analysis, H9C2 cells were cultured in 10 cm petri dishes. MHY1485, an agonist of mTOR, was applied to verified whether DHT can inhibit mTOR, sequentially lead to downregulation of NF-κB-mediated inflammatory response. PDTC, a NF-κB inhibitor, was set as the positive drug in vitro experiment.

### GFP-TFEB lentiviral vector transfection

The specific methods have been described in our previous study [26].

### Assessment of apoptosis by a Hoechst 33258 staining kit

H9C2 cells were fixed with ice-cold 4% paraformaldehyde for 20 min after washed with 0.1 mol/L sodium cacodylate buffer. Next, the cells were washed three times with 0.1 mol/L sodium cacodylate buffer before stained with Hoechst 33258 (Beijing Solarbio Science & Technology Co., Ltd., China) for 15 min in the dark. Finally, an inverted fluorescence microscope (Olympus; BX50-FLA; Japan) was applied to visualize the apoptotic cells.

### Immunofluorescence

Prior to incubation with primary antibody Cleaved caspase-3 (9664; Cell Signaling Technology, Germany) in a diluted concentration of 1:150 at 4 °C overnight, the paraffin-embedded sections need to be deparaffinized, inactivated with 0.3% hydrogen peroxide for 15 min and blocked with normal goat serum for 10 mins at room temperature, and then incubated with secondary antibody goat anti-rabbit IgG polyclonal (ab15007; Abcam, United States) for one hour at room temperature and dark place, followed by DAPI staining at room temperature for 5 min in the dark. Finally, sections were washed and fixed with antifade mounting medium. The optical microscope was used for photographing at 400 × magnification (Leica Microsystems GmbH).

The article "TFEB-NF-κB inflammatory signaling axis: a novel therapeutic pathway of Dihydrotanshinone I in doxorubicin-induced cardiotoxicity" was published in 2020. Journal: J Exp Clin Cancer Res.

H9C2 cells were grown on a laser confocal dish for the specified time, and then fixed with 4% paraformaldehyde for 15 min, followed by permeabilization (0.5% Triton X–100 in 0.1 mol/L sodium cacodylate buffer) for 20 min and blocked with normal goat serum for one hour. Later, cells were incubated with primary antibody overnight at 4 °C, followed by incubation with secondary antibody in the dark at room temperature for one hour. After being washed 3 times with PBS, cells were counterstained with DAPI (5 μg/mL) for 30 min. Images were then taken with a confocal microscopy.

### Western blot analysis

Protein samples were prepared and detected according to our previously described methods [26]. The antibodies we used were listed in Table 2.

**Table 2:** Primary antibodies used in western blot

Protein	Primary antibody
p-NF-κB	ab97726; Abcam, United States
NF-κB	CST8242; Cell Signaling Technology, Germany
TNF-α	ab205587; Abcam, United States
IL-8	ABM40268; Abbkine; United States
COX2	ab15191; Abcam; United States
p-IKKα/β	CST2697T; Cell Signaling Technology, Germany
IKKα	CST2682; Cell Signaling Technology, Germany
IKKβ	CST8943; Cell Signaling Technology, Germany
mTOR	CST2983; Cell Signaling Technology, Germany
p-mTOR	CST2971; Cell Signaling Technology; Germany
S6K1	ab9366; Abcam, United States
p-S6K1	ab2571; Abcam, United States
GAPDH	ab8245; Abcam, United States
rabbit IgG H&L	ab16284; HRP; Abcam, United States
mouse IgG H&L	ab97250; HRP; Abcam, United States
TFEB	13,372–1-AP; Proteintech; United States

### Data and statistical analysis

Statistical analyses were performed on GraphPad Prism software 6.0 (San Diego, CA, USA). All results were expressed as the mean ± SD. Comparisons between two groups were performed with the unpaired two-tailed t-test. Multiple comparisons were analyzed using ANOVA followed by Bonferroni-corrected post hoc test. The difference was considered statistically significant when *P* < 0.05. The statistical analysis abided the recommendations of the experimental design and analysis in pharmacology [27].

## Results

### Effects of DHT on cardiac function and structural alteration in DIC zebrafish model and in DIC mice model

Two days after DOX exposure, fish exhibited extensive pericardial edema and blood accumulation in tail (Fig. 1a). Microscopic examination revealed that the heart atrium was elongated, and the ventricle collapsed (Fig. 1a). By using a high-speed camera, we calculated the fractional shortening (FS) of the zebrafish hearts. The results showed that FS was dramatically decreased, resulting in reduced erythrocyte circulation within tail blood vessels (Fig. 1a, b, d). Moreover, both heart rate and survival rate were significantly reduced in DOX-treated zebrafish (Fig. 1c, e). DHT treatment protected against cardiotoxicity induced by DOX. It could up-regulate FS, promote blood flow in tail vein and rescue the survival rate in DIC zebrafish model.

The article "TFEB-NF-κB inflammatory signaling axis: a novel therapeutic pathway of Dihydrotanshinone I in doxorubicin-induced cardiotoxicity" was published in 2020. Journal: J Exp Clin Cancer Res.

**Fig. 1:** DHT improved cardiac function and protected against pathological injury in zebrafish and in mice. **a** Microscopic examination showed that DHT preserved the heart atrium, protected against extensive pericardial edema and blood accumulation in tail, and preserved the heart atrium. By using a high-speed camera, results and analysis showed that DHT increased FS values (**b**) and blood flow (**d**). DHT could improve heart rate (**c**) and survival rate (**e**). **f** M-mode echocardiography was assessed to detect cardiac function in each group. **g** Echocardiography data showed that DHT increased EF% and FS%, and decreased LVEDD and LVESD. **h** HE staining showed that DHT protected against the structural damage caused by DOX, scale bar = 20 μm. **i** Quantification of inflammatory cell infiltration (%) showed that DHT decreased the inflammatory cell rate. **j** Quantification of SOD and MDA levels in plasma. *N* ≥ 10 per group in zebrafish; *N* ≥ 5 per group in mice. All data were presented as means ± SD in triplicate. ^*^p < 0.05, ^**^p < 0.01, ^***^p < 0.001 is significantly different as indicated, for values in the DOX group

After four weeks of treatments, all mice were subjected to echocardiography to measure cardiac parameters, including LVEDD, LVESD, EF and FS (Fig. 1f, g). Echocardiography data showed that mice in the DOX group had significantly higher values of LVEDD and LVESD. After treatment with DHT, both of the values decreased. FS was reduced significantly in the DOX group as compared to that of the Saline group, indicative of reduced cardiac contractility. In contrast, FS of mice in the DOX + DHT group was significantly increased compared to mice in the DOX group, suggesting that left ventricular function was improved by DHT treatment. Besides, EF was also upregulated by DHT treatment. Hematoxylin and eosin (H&E) staining showed that the cardiac tissue was neatly arranged in the Saline group. A high number of infiltrated inflammatory cells and enlargement of the intercellular space could be observed in the DOX group, while treatment with DHT or Rapamycin rescued hearts from inflammatory cell infiltration and cellular injury (Fig. 1h, i). In addition, plasma MDA level was higher and SOD activity was lower in mice of the model group, as compared with those of the Saline group, while DHT treatment reversed the changes (Fig. 1j). Rapamycin had the similar effects to DHT (Fig. 1f-j).

The article "TFEB-NF-κB inflammatory signaling axis: a novel therapeutic pathway of Dihydrotanshinone I in doxorubicin-induced cardiotoxicity" was published in 2020. Journal: J Exp Clin Cancer Res.

### Effects of DHT on the accumulation of macrophages and M1 macrophages activation in DIC mice model and in LPS-stimulated RAW264.7 cells model

It is believed that recruitment of macrophages into the heart plays a pivotal role in the homeostasis of cardiac tissues [28]. Flow cytometry assay was applied to quantify the number of macrophages in cardiac tissue. CD11b + F4/80+ were used as biomarkers for macrophages. The results showed that the percentage of macrophages in the DOX group was significantly higher than that of the Saline group, indicating that circulating monocytes were mobilized to inflamed cardiac tissue and differentiated to macrophages in response to DIC. Treatment with DHT or rapamycin inhibited the recruitment of macrophages (Fig. 2a). Activated macrophages can be classified as either M1 (marked by CD86) or M2 (marker by CD206) macrophages. Our data showed a marked increase of M1 macrophages in DOX-treated mice, while treatment with DHT or rapamycin inhibited the activation of M1 macrophages (Fig. 2a). Besides, immunofluorescence assay showed that DHT suppressed the protein expressions of CD86 and F4/80 in mice. There was no difference of distribution of M2 macrophage among the four groups (Fig. 2b). Collectively, these data indicated that DHT exerted anti-inflammatory effect in DOX-stimulated mice probably by inhibiting activation of M1 macrophages.

**Fig 2:** DHT suppressed the activation of M1 macrophages in mice and in RAW264.7 cells. (A) Flow cytometry assay showed that DHT or Rapamycin reduced accumulation of macrophages and activation of M1 macrophages in mice. In (a), X-axis represents PE-Cy7 anti-CD11b and Y-axis represents APC anti-F4/80; in (b), X-axis represents PE anti-CD86 and Y-axis represents FITC anti-CD206. *N* ≥ 3 per group. ^*^p < 0.05, ^**^p < 0.01, ^***^p < 0.001 is significantly different as indicated, for values in the DOX group. **b** Immunofluorescence assay showed that DHT suppressed the protein expressions of CD86 and F4/80 in mice, scale bar = 20 μm. *N* = 3 per group. **c** DHT treatment for 24 h had no cytotoxic effect on RAW264.7 cells at the dosages of 10, 50 and 100 nM. *N* = 6 per group. **d** RAW 264.7 cells were stimulated with LPS (1 μg/mL) in the absence or presence of DHT (10, 50 and 100 nM) for 24 h and the releases of TNF-α and IL-1β in cell supernatants were detected by Elisa assay. N ≥ 5 per group. ^*^p < 0.05, ^***^p < 0.001 is significantly different as indicated, for values in the LPS group. **e** The protein expression of CD86 was detected by immunofluorescence assay. DHT suppressed the expression of CD86 in RAW264.7 cells, scale bar = 100 μm. *N* = 12 per group. **f** DHT reduced activation of M1 macrophages in LPS-stimulated RAW264.7 cells. N ≥ 3 per group. ^***^p < 0.001 is significantly different as indicated, for values in the LPS group. **g** DHT suppressed the nuclear localization of p-NF-κB in LPS-stimulated RAW264.7 cells, scale bar = 50 μm. *N* = 20 per group. All data were presented as means ± SD in triplicate.

The article "TFEB-NF-κB inflammatory signaling axis: a novel therapeutic pathway of Dihydrotanshinone I in doxorubicin-induced cardiotoxicity" was published in 2020. Journal: J Exp Clin Cancer Res.

To further investigate the effects of DHT on macrophages, LPS-stimulated RAW264.7 cell model was established. The CCK-8 assay showed that co-treatment of RAW264.7 cells with DHT (10, 50, and 100 nM) was nontoxic (Fig. 2c), and DHT could significantly decrease the LPS-induced expressions of TNF-α and IL-1β (Fig. 2d). Besides, immunofluorescence assay showed that DHT suppressed the expression of CD86 under LPS-stimulation (Fig. 2e). Flow cytometry assay furtherly proved that DHT could inhibit the activation of M1 macrophages (Fig. 2f). We also found that LPS-stimulation promoted expression and nuclear translocation of p-NF-κB (Fig. 2g). Collectively, the LPS-induced inflammatory responses were inhibited by DHT treatment. These in vitro results confirmed that the anti-inflammatory effect of DHT was partly exerted by suppressing activity of macrophages.

### Effects of DHT on NF-κB signaling pathway in DIC mice model and in DOX-stimulated H9C2 cells model

In mice, western blotting showed that the total NF-κB expression was unchanged among different groups. However, the expression of activated/phosphorylated NF-κB (p-NF-κB) increased in the heart tissue of DOX group. After treatment with DHT, the expression of p-NF-κB was reduced significantly (Fig. 3a). The expressions of downstream inflammatory genes activated by NF-κB were further detected. Levels of TNF-α, COX2 (Cyclooxygenase-2) and IL-8 in the DOX group were increased, as compared to the Saline group, whereas DHT treatment suppressed expressions of these downstream targets (Fig. 3a). To further evaluate the anti-inflammatory effects of DHT, the level of TNF-α was assessed. Content of TNF-α in homogenized fresh cardiac tissue was significantly up-regulated in the DOX group whereas treatment with DHT or rapamycin could effectively inhibit the expression of TNF-α (Fig. 3b). IHC of TNF-α was assessed and the result was consistent with Elisa result (Fig. 3c).

**Fig. 3:** DHT inhibited the production of pro-inflammatory cytokines mediated by NF-κB in mice and in cardiomyocytes. **a** Western blotting showed that DHT downregulated the expressions of activated NF-κB, TNF-α, COX2 and IL-8 in mice. *N* = 5 per group. All data were presented as means ± SD. ^*^p < 0.05, ^**^p < 0.01, ^***^p < 0.001 is significantly different as indicated, for values in the DOX group. **b** Quantification of TNF-α level in heart tissue. N = 5 per group. **c** IHC and quantitative results showed that DHT or Rapamycin suppressed the expression of TNF-α, scale bar = 20 μm. N = 5 per group. CCK-8 assay results showed the non-toxic range of concentration (**d**) and the protective concentrations (**e**). *N* = 12 per group. **f** Western blotting showed that DHT downregulated the expressions of activated NF-κB, TNF-α, COX2 in cardiomyocytes. N = 5 per group. All data were presented as means ± SD in triplicate. ^*^p < 0.05, ^**^p < 0.01, ^***^p < 0.001 is significantly different as indicated, for values in the DOX group

To further investigate the effects of DHT on NF-κB-mediated inflammation in myocardial cells, a DOX-stimulated H9C2 cell model was established [26]. Pre-treatment with 10 ~ 100 nM DHT for 24 h and co-treatment for 24 h proved to be effective (Fig. 3d and e). Besides, pyrrolidine dithiocarbamate (PDTC) was applied as a positive control drug, due to its direct inhibitory effects on NF-κB. Consistent with results in mice, western blotting results in cardiomyocytes showed that the expressions of p-NF-κB, TNF-α and COX2 were inhibited by DHT treatment, suggesting that DHT suppressed inflammation mediated by NF-κB signaling pathway (Fig. 3f).

The article "TFEB-NF-κB inflammatory signaling axis: a novel therapeutic pathway of Dihydrotanshinone I in doxorubicin-induced cardiotoxicity" was published in 2020. Journal: J Exp Clin Cancer Res.

### DHT inhibited inflammation by regulating mTOR-TFEB-NF-κB signaling pathway in DOX-stimulated cardiomyocytes

Recent studies reported that mTOR accumulation could induce inflammation [29, 30]. In this study, up-regulation of phosphorylated/activated mTOR was discovered in DOX-treated mice (Fig. 4a). The level of phosphorylated S6K, a downstream molecule reflecting the biological activity of mTOR, was also increased in DOX-treated mice (Fig. 4a). In mice treated with DHT, levels of phosphorylated mTOR and S6K were significantly reduced. Rapamycin showed similar effects in mice with DIC (Fig. 4a).

**Fig. 4:** DHT regulated mTOR-TFEB-NF-κB signaling pathway to ameliorate inflammation in DOX-stimulated cardiomyocytes. **a** Western blotting showed that DHT or rapamycin downregulated the expressions of phosphorylated mTOR and S6K in mice. N = 5 per group. All data were presented as means ± SD in triplicate. ^*^p < 0.05, ^**^p < 0.01, ^***^p < 0.001 is significantly different as indicated, for values in the DOX group. **b** Western blotting showed that with MHY1485 co-treatment, the effect of DHT on inflammation-related proteins including TNF-α and COX2 was abrogated in cardiomyocytes. N = 5 per group. All data were presented as means ± SD in triplicate. ^*^p < 0.05, ^**^p < 0.01, ^***^p < 0.001 is significantly different as indicated, for values in the DOX group. ^##^*p* < 0.01, ^###^*p* < 0.001 is significantly different as indicated, for values in the DOX + DHT group. **c** Cardiomyocytes were transfected with GFP-TFEB and results showed that co-treatment with MHY1485 abolished the effects DHT on the nuclear localization of TFEB, scale bar = 50 μm. N = 20 per group

To further confirm whether DHT inhibited inflammation through targeting mTOR, the mTOR agonist MHY1485 was utilized. Co-incubation with MHY1485 abolished the effects of DHT on expressions of p-NF-κB and the downstream pro-inflammatory genes, including TNF-α and COX2 (Fig. 4b). To investigate the effects of DHT on TFEB recruitment, H9C2 cells were transfected with a carried TFEB-GFP lentiviral vector (Lv). Results showed that DHT treatment could reduce the cytoplasmic localization and upregulate the nuclear recruitment of TFEB, while co-incubation with MHY1485 abolished this effect, indicating that TFEB is a mediator by which mTOR regulates NF-κB signaling pathway (Fig. 4c). Collectively, these results demonstrated that DHT ameliorated inflammation partly via mTOR-TFEB-NF-κB signaling pathway.

The article "TFEB-NF-κB inflammatory signaling axis: a novel therapeutic pathway of Dihydrotanshinone I in doxorubicin-induced cardiotoxicity" was published in 2020. Journal: J Exp Clin Cancer Res.

### DHT inhibited TFEB-IKK-NF-κB inflammatory signaling axis in cardiomyocytes

As compared to Lv-TFEB transfected cells, DOX treatment led to the decreased expression of TFEB in the nucleus (Fig. 5a). As compared to Lv-GFP transfected cells, DOX treatment upregulated the phosphorylation of NF-κB (Fig. 5a). It is worth noting that TFEB overexpression significantly reduced p-NF-κB expression and nuclear translocation, as compared to Lv-GFP transfected cells under DOX stimulation (Fig. 5a), furtherly confirming that TFEB could inhibit NF-κB activation and nuclear translocation. In addition, western blotting showed that phosphorylated level of IKKα/β and NF-κB in DOX-treated H9C2 cells was higher than that of cells without DOX treatment, accompanied by a reduced expression of nuclear TFEB (Fig. 5b-d). TFEB overexpression decreased levels of p-IKKα, p-IKKβ and p-NF-κB, suggesting that TFEB is an anti-inflammatory factor and may inhibit NF-κB activity by restraining IKK signaling pathway (Fig. 5b-d).

**Fig. 5:** DHT inhibited NF-κB transcriptional activity via TFEB-IKK signaling pathway. **a** Cardiomyocytes were transfected with Lentiviral vector (Lv) carrying GFP-TFEB to monitor the location of TFEB. Lv-GFP transfected cells were set as a negative control. Representative GFP fluorescence and immunofluorescence staining of p-NF-κB were shown under different treatment, scale bar = 100 μm. N = 20 per group. **b**, **c**, **d** Western blotting showed that DOX reduced the nuclear expression of TFEB and increased phosphorylated levels of IKKα/β and NF-κB, while DHT up-regulated the nuclear expression of TFEB. In particular, TFEB overexpression or DHT treatment down-regulated phosphorylated levels of IKKα/β and NF-κB. *N* = 3 per group. **e** Representative GFP-TFEB fluorescence and immunofluorescence staining of p-NF-κB under different treatment, scale bar = 50 μm. N = 20 per group. All data were presented as means ± SD in triplicate. *^*^p < 0.05, ^**^p < 0.01, ^***^p < 0.001

The effects of DHT on TFEB and IKKα/β were further explored. As shown in Fig. 5b, c and d, DHT treatment promoted nuclear localization of TFEB under DOX-stimulation. Meanwhile, after treatment with DHT, expressions of p-IKKα/β and p-NF-κB were reduced (Fig. 5b-d). Furthermore, DHT treatment inhibited nuclear localization of p-NF-κB (Fig. 5e). Inhibiting TFEB through application of mTOR agonist could abolish the effects of DHT on p-NF-κB (Fig. 4). Taken together, these data demonstrated that DHT inhibited NF-κB transcriptional activity via TFEB-IKK signaling pathway.

The article "TFEB-NF-κB inflammatory signaling axis: a novel therapeutic pathway of Dihydrotanshinone I in doxorubicin-induced cardiotoxicity" was published in 2020. Journal: J Exp Clin Cancer Res.

### DHT inhibited apoptosis of cardiomyocytes to facilitate the anti-inflammation effect

It is widely accepted that apoptosis is a potent inducer of inflammation [31]. The anti-apoptotic effects of DHT were further investigated. In vivo results showed that Cleaved caspase-3 expression in the left ventricle of heart was significantly increased in mice with DOX treatment, relative to mice in the Saline group (Fig. 6a). In mice treated with DHT or rapamycin, the expressions of Cleaved-Caspase 3 were reduced. Western blotting showed that DHT could also reduce expression of Bax and increase expression of Bcl-2 in mice treated with DOX, illustrating that DHT had anti-apoptotic effect (Fig. 6b).

**Fig. 6:** DHT inhibited apoptosis to facilitate the anti-inflammation effect. **a** The representative photomicrographs of a left ventricle section of the heart showed the expression of Cleaved caspase-3 under different treatment, scale bar = 20 μm. N = 5 per group. **b** Western blots detected the expressions of Bax and Bcl-2 proteins in heart tissues. N = 5 per group. **c** The results of Hoechst staining under different treatment, scale bar = 40 μm. N = 12 per group. **d** Western blots assessed the expressions of Bax and Bcl-2 proteins in H9C2 cells. N = 5 per group. All data were presented as means ± SD in triplicate. ^*^p < 0.05, ^**^p < 0.01, ^***^p < 0.001 is significantly different as indicated, for values in the DOX group. ^#^*p* < 0.05, ^##^*p* < 0.01 is significantly different as indicated, for values in the DOX + DHT group

Consistent with the in vivo experiment, in vitro study demonstrated that DHT significantly reduced the apoptotic rate, and regulated expressions of Bcl-2 and Bax in DOX-stimulated H9C2 cells (Fig. 6c, d). Interestingly, co-incubation with MHY1485 abolished the protective effects of DHT against apoptosis (Fig. 6c, d), indicating that the anti-apoptotic effect of DHT was partially mediated through mTOR pathway.

The article "TFEB-NF-κB inflammatory signaling axis: a novel therapeutic pathway of Dihydrotanshinone I in doxorubicin-induced cardiotoxicity" was published in 2020. Journal: J Exp Clin Cancer Res.

## Discussion

In the present study, in vivo and in vitro experiments were conducted to explore the protective effects of DHT against DIC and its underlying anti-inflammation mechanisms. The main findings are as follows: (1) DHT could improve cardiac functions evidenced by inhibiting the activation of M1 macrophages and excessive release of pro-inflammatory cytokines both in vivo (mouse and zebrafish) and in vitro (H9C2 and RAW264.7); (2) DHT could inhibit NF-κB-mediated inflammatory response via mTOR-TFEB pathway; (3) The TFEB-IKK-NF-κB axis plays a vital role in regulating DIC-related inflammation.

A growing body of evidence supports that DOX, as an effective chemotherapy drug, is a double-edged sword [32]. Indeed, irreversible injury to nontarget tissues often complicates cancer care by limiting therapeutic dosages of DOX and lowering the quality of patients’ life during and after DOX treatment [33]. Particularly, the heart is a preferential target of DOX and cardiotoxicity is one of the most severe side effects induced by DOX. Alterations in the administration of the drug, applications of liposomal DOX, and assistants with cardio-protective agents are the strategies that have been applied for the prevention or alleviation of cardiotoxicity. However, drugs that are commonly adopted to reduce DIC often have adverse effects. It is of great importance to explore novel therapeutic strategies with fewer side effects. A correlation between inflammation and adverse cardiovascular outcomes in DOX induced toxicity has been documented [34, 35]. Elevation of pro-inflammatory cytokines has been linked with worse DIC outcome in multiple studies [5]. Application of Chinese herbs that are able to mitigate inflammation without compromising the anti-tumor effect is of particular interest for the treatment of DIC.

Salvia miltiorrhiza Bunge is a well-known traditional herb with a long history of clinical application for the treatment of cardiovascular diseases [36, 37]. Its active ingredients have been widely investigated since last century [38]. For a long time, investigations into the bioactivities of DHT were mainly focused on cytotoxicity to various tumor cells [16, 39]. Emerged evidence pointed out that DHT has potential efficacy for curing cardiovascular diseases [40–42], however its anti-DIC effect, either in vivo or in vitro, has not been elucidated yet. The results of our study demonstrated that DHT treatment improved heart function in a DIC zebrafish model and in a DIC mouse model. It’s reported that DHT could play a therapeutic role in various inflammatory diseases, including atherosclerosis, allergic inflammation and colitis [43, 44]. Besides, DHT could modulate immune cell function, such as suppression of the release of cytokines [45]. To date, there have been no researches on the anti-inflammatory of DHT during application of DOX. Recruitment and activation of M1 macrophages have been reported to play a major role in DIC-related inflammation [34, 35]. Our in vivo *and* in vitro results showed that DHT could suppress accumulation of macrophages and activation of M1 macrophages under DOX-stimulation. Although it is still unclear as to the origin of heart macrophages, recent studies have suggested that these macrophages are derived from either the proliferation of resident macrophages or the differentiation of blood monocytes [46]. The in vitro results showed that expression of NF-κB and secretion of pro-inflammatory cytokines by macrophages were also inhibited by DHT. These data demonstrated that DHT could suppress inflammation by inhibiting activation of macrophages. Although pro-inflammatory cytokines are generally produced by activated macrophages, myocardial cells can also produce inflammatory agents through NF-κB-dependent pathway under pathological conditions. It’s noteworthy that NF-κB-mediated inflammatory response has been demonstrated as a pivotal pathway in DIC model [47, 48]. The involvement of pro-inflammatory cytokines driven by the activation of NF-κB can lead to the severe myocardial injury manifested by the dramatic reduction of the heart function [6, 49, 50]. Herein, the NF-κB pathway is believed to be one of the most attractive targets for DIC patients [48]. In current study, both in vivo and in vitro data showed that DHT suppressed cardiac levels of activated NF-κB as well as downstream inflammatory genes, including TNF-α, IL-8 and COX2 under DOX stimulation. The effect of DHT on the upstream regulative pathway was further investigated.

The article "TFEB-NF-κB inflammatory signaling axis: a novel therapeutic pathway of Dihydrotanshinone I in doxorubicin-induced cardiotoxicity" was published in 2020. Journal: J Exp Clin Cancer Res.

The mTOR protein is a serine/threonine kinase that regulates a variety of cellular functions. Update studies suggest that it is also an important regulator of inflammation responses. A number of studies have indicated that pharmacological inhibition of mTOR can provide anti-inflammatory protection [20, 30, 51]. Rapamycin is a specific inhibitor of mTOR and was applied as positive control drug in this study. Intriguingly, rapamycin dramatically improved cardiac functions and inhibited inflammatory response in DIC models. DHT had similar inhibitory effect on mTOR as rapamycin, providing evidence that mTOR is a potential pharmacological target of inflammation response in DIC. Previous study reported that mTOR inhibitors augmented the anti-inflammatory activities of regulatory T cells and reduced the production of pro-inflammatory cytokines by macrophages [52]. In this study, we focused primarily on the inflammatory regulatory effects and mechanisms of mTOR signaling pathway in cardiomyocytes. The mTOR agonist, MHY1485, was applied to DOX-stimulated H9C2 cells. After co-incubation with MHY1485, the effects of DHT on NF-κB, TNF-α, COX2 and nuclear TFEB were abrogated, suggesting that the protective mechanism of DHT on inflammatory response is mainly mediated by mTOR-NF-κB signaling pathway, moreover, TFEB plays pivotal roles in this signaling pathway.

TFEB has been recently identified as serving critical and diverse roles in immune systems [8]. Then, to verify how the TFEB participates in mTOR-NF-κB pathway, loss/gain of the function of TFEB were performed. We found that DOX treatment reduced the expression of nuclear TFEB, and up-regulated phosphorylation of IKKα/β and NF-κB, suggesting that there might be a link between TFEB and NF-κB activation. When H9C2 cells were transfected with lentiviral vector carrying GFP-TFEB, TFEB overexpression downregulated the expressions of activated IKKα/β and NF-κB, further indicating that the IKK-NF-κB signaling axis is directly inhibited by TFEB. Targeting TFEB using pharmacological agents may, therefore, hold great promise against cardiac inflammatory complications. Intriguingly, DHT treatment promoted nuclear localization of TFEB and downregulated the expressions of p-IKKα/β and p-NF-κB, while inhibiting TFEB through application of mTOR agonist could abolish the effects of DHT on p-NF-κB. These data demonstrated that DHT inhibited NF-κB transcriptional activity via TFEB-IKK signaling pathway. Taken together, our data offered the evidence that DHT inhibited NF-κB-mediated inflammatory response through mTOR-TFEB-IKK signaling pathway.

In the present study, we also investigated the anti-apoptotic effects of DHT. Though apoptotic cells could trigger or potentiate inflammation, the underlying mechanism remains to be clarified [31]. In consistent with previous reports [53–55], we found that DOX could induce apoptosis and DHT has anti-apoptotic effects. We further explored the role of mTOR in apoptosis [56]. Intriguingly, co-incubation of cells with mTOR agonist abolished the inhibitory effects of DHT on apoptosis, suggesting that DHT exerted anti-apoptosis effects via mTOR signaling pathway. The mTOR signaling may serve as the co-regulator of both inflammatory and apoptotic pathway. The underlying molecular mechanism warrants further investigation.

The article "TFEB-NF-κB inflammatory signaling axis: a novel therapeutic pathway of Dihydrotanshinone I in doxorubicin-induced cardiotoxicity" was published in 2020. Journal: J Exp Clin Cancer Res.

## Conclusion

For the first time, our research demonstrated TFEB-IKK-NF-κB inflammatory signaling axis as a novel therapeutic pathway for DIC. DHT can be applied as a potential agent for the anti-inflammation treatment of DIC via mTOR-TFEB-NF-κB signaling pathway. This study provides the possibility of adjuvant therapies that protect the heart as well as improving anti-tumor effects. In addition, it will be informative to explore whether DHT’s cardioprotective effects could extend to other modes of heart injury, such as ischemia or other cardiotoxic chemotherapies.

## Data Availability

The datasets used and/or analysed during the current study are available from the corresponding author on reasonable request.

## Abbreviations

CMC: Carboxymethylcellulose
COX2: Cyclooxygenase-2
DAB: Diaminobenzidine
DHT: Dihydrotanshinone I
DIC: Doxorubicin-induced cardiotoxicity
DMEM: Dulbecco’s Modification of Eagle’s Medium
DMSO: Dimethyl sulfoxide
DOX: Doxorubicin
dpf: Day postfertilization
EF: Ejection fraction
FS: Fraction shortening
HE: Hematoxylin-Eosin
IκB: Inhibitor of NF-κB
IKKs: IκB kinases
IL-8: Interleukin 8
LVEDD: Left ventricular end-diastolic dimension
LVEDV: Left ventricular end-diastolic volume
LVESD: Left ventricular end-systolic dimension
LVESV: Left ventricular end-systolic volume
MDA: Malondialdehyde
mTOR: Mammalian target of rapamycin
NF-κB: Nuclear factor-κB
PBS: Phosphate buffer saline
PDTC: Pyrrolidine dithiocarbamate
Rapa: Rapamycin
SOD: Superoxide dismutase
SPF: Specific Pathogen Free
TCM: Traditional Chinese medicine
TFEB: Transcription factor EB
TNF-α: Tumor necrosis factor-α
